This article has been retracted.

# A Clinical Study on the Treatment of Children's Short Stature with Auxiliary Comprehensive Management Combined with Growth Patch

**DOI:** 10.1155/2021/7142006

**Published:** 2021-10-27

**Authors:** Haiying Feng, Weizhu Zhao, Huijun Yu, Guanfu Wang, Qunhong Wang

**Affiliations:** ^1^Department of Pediatrics, Taizhou Hospital of Zhejiang Province Affiliated to Wenzhou Medical University, Taizhou 318050, Zhejiang, China; ^2^Department of Urology, Taizhou Hospital of Zhejiang Province Affiliated to Wenzhou Medical University, Taizhou 318050, Zhejiang, China; ^3^Department of Traditional Chinese Medicine, Taizhou Hospital of Zhejiang Province Affiliated to Wenzhou Medical University, Taizhou 318050, Zhejiang, China

## Abstract

**Objective:**

To explore the clinical effect of auxiliary comprehensive management combined with growth patch in the treatment of childhood idiopathic short stature (ISS).

**Methods:**

From September 2017 to December 2019, 120 children with ISS who met the selection criteria were collected. Random number table method divided them into 2 groups: one group was given auxiliary comprehensive management and recorded as the routine group (*n* = 60), and the other group was given auxiliary comprehensive management and combined growth patch treatment and recorded as the combination group (*n* = 60). The course of treatment was 12 months. The effects of the two methods on children's height, bone age, body weight, and insulin-like growth factor (IGF)-1 and IGF-binding protein (IGFBP)-3 levels were compared.

**Results:**

There was no statistical difference between the two groups in baseline height, genetic height, baseline bone age, baseline body weight, and body weight before and after treatment (*P* > 0.05). After treatment, the heights of the two groups were higher than before for the same group, the height growth values and predicted adult height of the combination group were higher than those of the routine group, and the predicted adult height of the combination group was higher than the genetic height of the same group (*P* < 0.001). There was no statistical difference in IGF-1 and IGFBP-3 levels before treatment between the two groups (*P* > 0.05). The levels of IGF-1 and IGFBP-3 after treatment in the two groups were higher than those in the same group before treatment, and the combination group was higher than that in the routine group (*P* < 0.05).

**Conclusion:**

On the basis of auxiliary comprehensive management, combined with growth patch for the treatment of children with ISS, it can effectively increase the height of the children, improve the levels of serum IGF-1 and IGFBP-3, and have significant clinical effects, which is beneficial to the healthy growth of the children.

## 1. Introduction

Short stature in children refers to patients whose height is significantly shorter than the average height of the normal population by 2 standard deviations (−2SD) or lower than the third percentile (−1.88sd) among individuals of the same race, gender, and age under normal living standards, and the bone maturity is evaluated according to bone age and less than 2 years behind the actual age [1, 2]. According to statistics, the rate of growth retardation in children in my country is as high as 9.9%, but the overall treatment rate is less than 1%. There are many factors that cause the disease. Growth hormone (GH) deficiency, hypothyroidism, idiopathic shortness, intrauterine growth retardation, and IGF deficiency are the five main causes of short stature in children [3–6]. In addition to the disease that can cause children with short stature, children may be accompanied by mental and psychological disorders, introverted personality, lack of cognition, activity, and social skills [7, 8]. For the treatment of short stature in children, modern medicine usually adopts subcutaneous injection of GH, but the response of GH treatment to individuals is difficult to predict, and it has brought heavy economic and psychological burdens to many families [9–11].

Short stature belongs to the name of modern medicine, and according to its clinical manifestations, it can be classified into the category of “five delays” in Traditional Chinese Medicine. The main responsibility is the deficiency of the spleen and kidney, and it is also related to the liver. The kidney is the congenital foundation, which controls the growth of bone marrow; the spleen is the foundation of acquired nature, which controls the metaplasia of qi and blood. The growth and development of the human body depend on the nourishment of the kidney essence and the transport and transformation functions of the spleen. Deficiency of kidney essence and lack of the source of bone marrow metaplasia will slow the growth of bones, leading to short stature, insufficient spleen source and viscera lose nourishment, resulting in growth retardation. In addition, the liver stores blood and controls the dredging, corresponding and relating to the tendons and claws of the body. If the liver blood is sufficient, the muscles and bones will be nourished, and if the liver blood is deficient, the muscles and bones will be dystrophic, leading to slow growth and short stature.

Based on the above theory, Chinese medicine has accumulated rich clinical experience in the use of pediatric massage, acupoint application, and other therapies to prevent and treat children with short stature, and there are no toxic side effects. In recent years, our department uses traditional Chinese medicine and trace elements as raw materials to make a self-made growth patch for children. The effect of the drug is penetrated through local acupoint pressing, and the effect of the growth patch on the levels of serum IGF-1 and IGFBP-3 in children with ISS has been tested. It is hoped to discover the clinical effect and mechanism of action of the combined growth patch in the treatment of children's short stature on the basis of auxiliary comprehensive management. See the report below.

## 2. Materials and Methods

### 2.1. General Data

From September 2017 to December 2019, 120 children with ISS who met the selection criteria were collected. Random number table method divided them into 2 groups: one group was given auxiliary comprehensive management and recorded as the routine group (*n* = 60), and the other group was given auxiliary comprehensive management and combined growth patch treatment and recorded as the combination group (*n* = 60). There was no statistical difference between the baseline information in Table 1 of the routine group and the combined group, and they were comparable (*P* > 0.05).

### 2.2. Inclusion Criteria [12]

① Age 5∼12 years old; ② those whose height is lower than two standard deviations or below the 3rd percentile of the normal reference value of the same age, sex, region, and race; ③ the body length at birth was within the normal range of body length at the same gestational age, and the body mass and body proportions were normal; ④ the chromosome examination was normal and the peak GH was ≥10 *μ*g/L; ⑤bone age film showed that the epiphysis had not been closed; ⑥ those with normal or delayed bone age; ⑦ those with normal thyroid function, liver, kidney, heart, and lung function; ⑧ children and their family members who had informed consent to this study and had good compliance.

### 2.3. Exclusion Criteria

① Those with GH deficiency (peak GH < 10 *μ*g/L), hypothyroidism and other endocrine diseases; ② those with pituitary diseases, genetic metabolic diseases, skeletal development disorders, malnutrition, eating disorders, precocious puberty, and various chronic systemic diseases; ③ those with abnormal intellectual development or severe mental or emotional disorders; ④ those who were allergic to the drugs used in this study or had skin allergies; ⑤ those who had recently taken other drugs that affect serum IGF-1 and IGFBP-3 levels; ⑥ those who were unwilling to cooperate with this study.

### 2.4. Treatment Methods

During the treatment period, the two groups of children all implemented auxiliary comprehensive management. Specifically as ① diet management: balanced nutrition, prevent picky eaters and obesity, prevent excessive intake of protein and oil, moderate intake of coarse grains and fiber foods, prevent premature sexual development, eat less off-season fruits and vegetables, avoid health products, and eat carefully foods that may contain hormones or drugs that enhance immunity; ② sleep management: ensuring adequate sleep for 10 hours a day, and ensuring entering deep sleep before 22:00 every day; ③ sports management: according to the children's hobbies, developing a reasonable exercise plan, such as running, playing ball, skipping rope, and swimming, ensuring more than 30 minutes of exercise time per day, and adjusting the exercise intensity according to the children's physical fitness, avoiding excessive exercise and sports injuries; ④ medication management: appropriate supplementation of conventional nutrients such as calcium, vitamin B, and trace elements; ⑤ psychological management: strengthening the interaction and communication with the children, creating a warm and comfortable growth environment for the children, giving timely psychological counseling to the children with inferiority complex, nervousness and other bad psychology, protecting the self-esteem of the children, so that it actively cooperates with doctors to complete various treatments and examinations; ⑥ establishing a WeChat group to implement dedicated management, supervision and reminders to ensure good sleep and exercise time for children. When problems occurred during treatment, they would be resolved in time. Intervention was for 12 months.

On this basis, the combination group was combined with growth patch therapy. The growth patch was configured by the Department of Traditional Chinese Medicine in this hospital. The ingredients of the medicine included *Codonopsis*, *Astragalus*, Kumble, Oysters, Borneol, Menthol, Licorice, Vitamin E, Vitamin A, Camphor, Salicylic acid, and Zinc preparations. Selection of points: Shenque, Zusanli, Yongquan, Guanyuan, and Shenshu. Method and course of treatment: the above-mentioned drugs were ground into fine powder together, sieved, mixed evenly, and bottled for later use. Take out 1∼2 g of each application to make a paste pill and apply it on the above-mentioned acupuncture points, and finally fix it with a medical patch. After application, the above-mentioned acupoints were properly massaged through the growth patch for 3∼5 min to promote the absorption of the drug effect. 1 time/week, 2∼4 h/time, 3 months was 1 course of treatment, 4 courses of treatment.

### 2.5. Observation Indicators

1. Growth indicators: The baseline height, genetic height, height after 12 months of treatment, height growth value, and predicted adult height were compared between the two groups. Boy's genetic target height = (father's height + mother's height + 13)/2 (cm); Girl's genetic target height = (father's height + mother's height − 13)/2 (cm); predicted adult height (using Tanner-Whitehouse 3 method). According to the bone age value evaluated by the Chinese children and adolescent bone age evaluation software, the corresponding prediction formula was used for prediction. The bone age and body weight of the two groups before and after treatment were compared. The bone age of all children was estimated by taking left-hand X-rays.
2. Serological indicators: Before and after treatment, two groups of peripheral fasting blood were drawn to detect serum IGF-1 and IGFBP-3 levels. Method: 6 mL of venous blood was drawn in the morning, centrifuged at 2800 r/min for 8 min, and the supernatant was separated and placed in a refrigerator at −30°C for testing. All detections were carried out by automatic immunochemiluminescence method. The kit was provided by Shanghai Keyuan Biotechnology Co., Ltd., and the analyzer used was the Beckman Coulter UniCel Dx1800 automatic chemiluminescence immunoassay analyzer.

### 2.6. Statistical Methods

Data analysis was processed by SPSS 22.0 software. The measurement data was expressed as ($\bar{x}\pm s$), and *t*-test analysis was used for comparison. The count data was expressed as (%), and *χ*^2^-test analysis was used for comparison. *P* < 0.05 indicated that the difference was statistically significant.

## 3. Results

### 3.1. Comparison of Height Differences between the Two Groups

The baseline heights of the routine group and the combination group were (107.06 ± 4.65) and (107.12 ± 4.23) cm, respectively; the genetic heights were (156.74 ± 4.68) and (156.51 ± 4.87) cm, respectively. After treatment, the heights of the routine group and the combination group were (111.86 ± 4.20) and (115.97 ± 4.85) cm, respectively; the height growth values were (3.85 ± 1.34) and (7.89 ± 1.54) cm, respectively; the predicted adult heights were (156.84 ± 4.32) and (165.60 ± 5.28) cm, respectively. There was no statistical difference in baseline height and genetic height between the two groups (*P* > 0.05). After treatment, the heights of the two groups were higher than before the same group, the height growth values and predicted adult height of the combination group were higher than those of the routine group, and the predicted adult height of the combination group was higher than the genetic height of the same group (*P* < 0.001) (Figure 1).

### 3.2. Comparison of the Differences in Bone Age between the Two Groups

The baseline bone ages of the routine group and the combination group were (8.97 ± 1.52) and (9.03 ± 1.49) years old, respectively (*P* > 0.05). After treatment, the bone ages of the routine group and the combination group were (9.86 ± 1.75) and (9.98 ± 1.80) years old, respectively (*P* > 0.05). The bone age after treatment in the two groups was higher than that before treatment in the same group (*P* < 0.05) (Figure 2).

### 3.3. Comparison of the Differences in Body Weight between the Two Groups

The baseline body weights of the routine group and the combination group were (28.63 ± 9.85) and (27.96 ± 10.12) kg, respectively (*P* > 0.05). After treatment, the body weights of the routine group and the combination group were (29.28 ± 10.01) and (30.62 ± 9.94) kg, respectively (*P* > 0.05). There was no statistical difference between the two groups of body weight before and after treatment (*P* > 0.05) (Figure 3).

### 3.4. Comparison of Serum IGF-1 and IGFBP-3 Levels between the Two Groups

Before treatment, the levels of IGF-1 in the routine group and the combination group were (97.52 ± 11.60) and (97.81 ± 12.03) ng/mL, respectively (*P* > 0.05); the levels of IGFBP-3 were (3.17 ± 0.45) and (3.20 ± 0.46) *μ*g/mL, respectively (*P* > 0.05). After treatment, the IGF-1 levels of the routine group and the combination group were (258.69 ± 40.64) and (357.50 ± 50.47) ng/mL, respectively; the IGFBP-3 levels were (4.96 ± 0.45) and (6.39 ± 0.44) *μ*g/mL, respectively. The levels of IGF-1 and IGFBP-3 after treatment in the two groups were higher than those in the same group before treatment, and the combination group was higher than the routine group (*P* < 0.001) (Figure 4).

## 4. Discussion

Short stature is one of the more common diseases in pediatrics. ISS is the most common cause of the disease, accounting for about 60–80% of all children with short stature. ISS refers to a growth and development disorder caused by unknown or genetic reasons, the child's GH level is normal, and there are no systemic diseases, endocrine diseases, nutritional disorders, or chromosomal abnormalities, which is an exclusive diagnosis [13]. Nutritional support, exercise therapy, and drug intervention are effective ways to treat short stature. Among them, drug therapy is the most effective. Common drugs include recombinant human GH (rhGH), long-acting rhGH, and rhIGF-1 [14]. All have the benefit of improving lifelong high, but their curative effect is affected by the child's age, etiology, genetics and treatment course, etc. and also has the risk of inducing abnormal glucose metabolism, hypothyroidism, benign intracranial hypertension, scoliosis, pigmented moles, enlarged hands and feet, and tumors [15]. Therefore, it is necessary to comprehensively consider the long-term efficacy, safety, and economic benefits of the drug in clinical application and carefully evaluate and select it.

Traditional Chinese medicine is a treasure of the Chinese nation, and “holistic concept” and “dialectical treatment” are its characteristic theories. In recent years, the research of traditional Chinese medicine in the prevention and treatment of short stature in children has attracted more and more attention. The theory of traditional Chinese medicine believes that the five internal organs of children have the physiological characteristics of “the heart and liver are surplus, but the lungs, spleen and kidney are often insufficient.” The growth of children's body and the development of wisdom depend on the nourishment of the kidneys, spleen, and stomach. According to modern research, the incidence of ISS is mostly related to heredity, and most of the children are accompanied by decreased expression of IGF-1 and IGFBP-3 and insufficient nutritional intake; as a result, growth is slowed down, the daily demand for nutrients is reduced, and the nutritional intake of children is reduced, and it forms a vicious circle with the slowdown of the body's growth, which will inevitably lead to short stature and underweight problems [16, 17]. This is consistent with the view of traditional Chinese medicine theory that the kidney stores essence, which provides the necessary material basis for various functions of the human body, and the child's congenital deficiency of essence and blood affects the growth and development and leads to short stature; the spleen and stomach are the foundation of the acquired, digesting, absorbing, and spreading various nutrients needed for life activities; when the spleen and stomach have loss of transport, it will lead to anorexia, vomiting, diarrhea, stagnation or malnutrition in children, and other diseases, affecting nutrition intake, and then delayed development. In addition, the growth and development of children also depend on the ascending function of the liver of “dominate the catharsis and regulate the activity of qi.” Liver qi communicates with spring qi, which is manifested as growth and vitality. It can be seen that Traditional Chinese Medicine also has unique advantages in the prevention and treatment of short stature in children starting from the “liver.” Some scholars also believe that Chinese medicine should fully integrate the growth and development of children with their own laws in treating children with short stature. For children with short stature under 2 years old, the spleen and stomach should be regulated; for children 2–10 years old, the liver and spleen should be regulated; and the liver and kidney should be emphasized during adolescence.

Based on the above theory, this study used growth patch to treat children with ISS on the basis of routine auxiliary comprehensive management. As a result, there was no statistical difference in baseline height and genetic height between the two groups, but after treatment, the heights of the two groups were higher than before for the same group, and the height growth values and predicted adult height of the combination group were higher than those of the routine group, and the predicted adult height of the combination group was higher than the genetic height of the same group. This suggests that, on the basis of auxiliary comprehensive management, the combined application of growth patch is an effective way to effectively promote the growth rate of children without accelerating bone age healing.

In this study, the growth patch was made of *Codonopsis*, *Astragalus*, Kumble, Oysters, Borneol, Licorice, Vitamin E, Vitamin A, and Zinc preparations. Among them, *Codonopsis* and *Astragalus* enter the spleen and lung meridian, can nourish the spleen and lung, and nourish blood and body fluid. *Codonopsis* glycosides, *Codonopsis pilosula* polysaccharides and trace elements, and other pharmacological components can enhance immunity and hematopoietic function and improve learning memory and digestive functions [18]; the pharmacological components of *Astragalus* extract can improve the material metabolism of the endocrine system (hypothalamus-pituitary-protein synthesis, lowering blood sugar) and can increase the expression of IGF to promote the growth rate of rats [19]. Kumble enters the liver and kidney meridians, and the iodine contained in it plays a key role in the synthesis and secretion of thyroid hormones. Thyroid hormone is a key hormone that regulates the metabolism of energy substances required for the growth and development of the body and is of great significance to the metabolism, growth, and development of the human body [20]. When iodine is deficient, it can cause different degrees of mental retardation, neurological disorders, physical development disorders, and dry skin and hair in adolescents and children. Therefore, proper supplementation of iodine in children with ISS not only is beneficial to their physical growth, but also helps prevent the lack of intellectual development [21]. It is reported that the secretion of GH that affects height growth during sleep is about three times that of the waking state. In the growth patch, Oysters enter the liver and kidney meridians, can nourish yin and yang, calm the nerves, improve children's sleep, and facilitate the normal secretion of GH in children. Oysters also contain calcium carbonate, calcium phosphate, calcium sulfate, iron, zinc, manganese, copper, and other trace elements and amino acids [22]. According to research, the levels of calcium, zinc, and iron in the whole blood of children with short stature are significantly lower than those of normal healthy children [23]. In the growth patch, the preparation of Chinese medicinal materials rich in trace elements and zinc preparations can effectively supplement the lack of trace elements in children with short stature and improve the nutritional status. Borneol is aromatic and refreshing, attracting drugs ascending. It can help the shared drugs to be absorbed through the skin and improve the in vivo pharmacokinetics of the shared drugs. Licorice harmonizes the properties of various drugs and can nourish the spleen and stomach. Vitamin E and Vitamin A are fat-soluble vitamins. According to previous reports, the main clinical manifestation of children with short stature is short stature, followed by abnormal metabolism and delayed bone maturation; when children have abnormal fat metabolism, it is easy to cause absorption and metabolism disorders of fat-soluble vitamins [24]. In this study, regarding the formulation of vitamin E and vitamin A in the growth patch, the former can regulate the expression of GH and IGF and then improve body weight and growth rate [25]; the latter can promote cell differentiation and maturation, induce growth acceleration, and improve appetite [26, 27]. In addition, this study performed acupoint pressing on the children's application sites—Shenque, Zusanli, Yongquan, Guanyuan, and Shenshu. On the one hand, the proper massage technique helps fully penetrate the drug ingredients. On the other hand, the application of Shenque and Zusanli helps invigorate qi and invigorate the spleen and promote the movement of spleen and stomach; the application of Yongquan, Guanyuan, and Shenshu can invigorate the kidney qi and solid foundation and strengthen the waist and knees. The synergistic effect of the above-mentioned drugs and acupoint massage can promote the body's metabolism, improve sleep and appetite, promote the blood circulation of the epiphysis, and finally achieve the purpose of increasing height. At the same time, the above drugs may also promote the functional activities of the hypothalamus-pituitary-growth axis and osteoblasts, ultimately improving bone development and enhancing children's physical fitness and disease resistance.

IGF, also known as somatomedin, is a type of cell growth-promoting polypeptide whose amino acid sequence and function are similar to those of insulin, including IGF-1 and IGFBP-3 [28]. At present, more and more evidences show that linear growth in human height is regulated by the growth hormone-releasing hormone (GHRH)-GH-IGF1 axis [29]. Among them, GH is mainly synthesized and secreted by the anterior pituitary gland, which plays an important role in growth regulation and normal human growth, and regarding its deficiency or abnormal molecular structure and receptors, it can lead to growth disorders. Its most important growth effect may be achieved through serum IGF1, and therefore children with short stature tend to have lower serum IGF-1 levels than normal children of the same age and gender. In addition, serum IGFBP-3, the most abundant IGF-binding protein in blood after birth, binds to IGFs, prevents their degradation, facilitates IGF transport in various parts of the body, and modifies the structure of IGFs so as to alter the interaction between IGFs and their specific receptors. It is also GH-dependent and correlates with the amount of GH secretion, so its measurement is also useful for the detection of abnormal GH secretion. In this study, we use growth patch to treat children with ISS and detect the changes of the above factors. The results showed that the levels of IGF-1 and IGFBP-3 after treatment in the two groups were higher than those in the same group before treatment, and the combination group was higher than that in the routine group. This suggests that the growth patch's mechanism of improving ISS may be related to the regulation of serum IGF-1 and IGFBP-3 levels in the body.

In summary, On the basis of auxiliary comprehensive management, combined with growth patch for the treatment of children with ISS, it can effectively increase the height of the children, improve the levels of serum IGF-1 and IGFBP-3, and have significant clinical effects, which is beneficial to the healthy growth of the children.

## Figures and Tables

**Figure 1:** Comparison of height differences between the two groups ($\bar{x}\pm s$, cm). (a) Comparison of height between the two groups before and after treatment. (b) Comparison of height growth value, genetic height, and predicted adult height between the two groups. ^*∗*^comparison with the same group before treatment, *P* < 0.001; ^#^comparison with the routine group after treatment, *P* < 0.001; ^&^comparison with genetic height of the same group, *P* < 0.001.

**Figure 2:** Comparison of the differences in bone age between the two groups ($\bar{x}\pm s$, years old). ^*∗*^Comparison with the same group before treatment, *P* < 0.05.

**Figure 3:** Comparison of the differences in body weight between the two groups ($\bar{x}\pm s$, kg).

**Figure 4:** Comparison of serum IGF-1 and IGFBP-3 levels between the two groups. (a) IGF-1 level. (b) IGFBP-3 level. ^*∗*^Comparison with the same group before treatment, *P* < 0.001; ^#^comparison with the routine group after treatment, *P* < 0.001.

**Table 1:** Comparison of baseline information between the two groups.

Category	Routine group (*n* = 60)	Combination group (*n* = 60)	*χ* ^2^/*t*	*P*
Gender (boy/girl)	33/27	36/24	0.307	0.580
Age (years old)	8.41 ± 1.82	8.74 ± 1.89	0.974	0.332
Height (cm)	107.06 ± 4.65	107.12 ± 4.23	0.074	0.941
Bone age (years old)	8.97 ± 1.52	9.03 ± 1.49	0.218	0.828
Body weight (kg)	28.63 ± 9.85	27.96 ± 10.12	0.367	0.714

## Data Availability

The primary data to support the results of this study are available at reasonable request to the corresponding author.
